RETRACTED

# miR-29b Regulates Lung Cancer Progression by Downregulating FEM1B and Inhibiting the FOX01/AKT Pathway

**DOI:** 10.1155/2022/3110330

**Published:** 2022-08-14

**Authors:** Huanrong Zhang, Rong Wang, Qiuhua Deng

**Affiliations:** ^1^Department of Thoracic Surgery, Meizhou People's Hospital (Huangtang Hospital), Meizhou Academy of Medical Sciences, Meizhou, China; ^2^The Translational Medicine Laboratory, The First Affiliated Hospital of Guangzhou Medical University, Guangzhou, China

## Abstract

**Purpose:**

Lung cancer is a relatively common type of cancer, and the incidence rate has been on the rise in recent years. MicroRNAs are a class of endogenous small RNA molecules, which are essential for the posttranscriptional regulation of genes. miR-29b is closely related to the occurrence and development of tumors, including prostate cancer, colon cancer, and breast cancer. However, few studies have been performed to explore the expression and pathway of miR-29b in non-small-cell lung cancer (NSCLC).

**Methods:**

Using bioinformatics analysis, we found that patients with low relative expression of the miR-29b gene have a low long-term survival rate. The results of in vitro research showed that when miR-29b expression was upregulated, the invasion, migration, and proliferation of A549 and NCI-H-1792 cells was inhibited, and the apoptosis was accelerated.

**Results:**

The results showed that FEM1B is a miR-29b target gene, and the expressions of FEM1B and miR-29b were negatively correlated. Like the upregulation of miR-29b expression, silencing the FEM1B expression could also impair the invasion, migration, and proliferation abilities of A549 and NCI-H-1792 cells. When FEM1B expression was restored, the inhibitory effect of miR-29b could be reversed. Reverse transcription-polymerase chain reaction (RT-PCR) and western blot (WB) analysis showed that overexpression of miR-29b could inhibit the expression of FEM1B, AKT, vascular endothelial growth factor (VEGF), and Sirt3 in A549 and NCI-H-1792 cells and upregulate the expression of FOXO1 protein.

**Conclusion:**

The results of this study indicate that miR-29b inhibits the proliferation and deterioration of NSCLC cells by targeting FEM1B and inhibiting the activation of the FOXO1/AKT pathway. miR-29b may become a new target for the clinical diagnosis and treatment of lung cancer, and it is expected to become a new inhibitor of NSCLC.

## 1. Introduction

Lung cancer is a common disease entity in today's society. It has high morbidity and high mortality [1–3]. The incidence of lung cancer accounts for 11.6% of the global cancer [4]. About 1.8 million people are diagnosed with lung cancer every year in the world and 1.6 million people die of lung cancer [5]. Lung cancer is divided into non-small-cell lung cancer (NSCLC) and small cell lung cancer on the basis of histological classification. The NSCLC accounts for 80% of the total lung cancer incidence [6, 7]. Although the medical level has continuously improved in recent years and the treatment and diagnosis methods have constantly updated, the cure rate of NSCLC is not ideal. According to surveys, the long-term survival rate of NSCLC in Europe is only 10% [8]. NSCLC is mostly diagnosed in the middle and late stages, and it is not easy to detect this entity during early screening. This is also one of the most important reasons for the unsatisfactory treatment effect. NSCLC lacks markers for early diagnosis and targeted therapy, which is also the main factor for the poor prognosis and low long-term survival rate of patients with NSCLC.

RETRACTED

MicroRNAs are a type of endogenous noncoding RNA with regulatory functions [9, 10]. By regulating the expression of gene transcription proteins, they play an important role in the processes of cell proliferation, differentiation, and apoptosis. Due to its wide range of functions, miRNA has become a potential biological standard and targeted therapy site in the occurrence of tumors [11–14]. Studies have shown that miRNA can be used as a specific target in the diagnosis and treatment of lung cancer [15–18]. Similarly, miR-29b is closely related to the occurrence and development of lung cancer [19], but its mechanism and potential role in lung cancer are not yet clear.

This study was aimed at determining the role of miR-29b on regulating the lung cancer progression and the underlying mechanism, which demonstrated that FEM1B and the FOX01/AKT pathway participated in this progress.

## 2. Materials and Methods

### 2.1. Test Materials and Cell Culture

A549, Calu-1, Calu-6, HCC827, NCI-H-1792, and BEAS-2B were purchased from Shanghai Institute of Biochemistry and Cell Biology (Shanghai, China). A549, Calu-1, Calu-6, HCC827, NCI-H-1792, and BEAS-2B cells were cultured in Dulbecco's Modified Eagle Medium (DMEM), 10% fetal bovine serum (Gibco, Waltham, MA USA), and 1% double antibody (Gibco, Waltham, MA, USA) in a cell culture incubator at 37°C and 5% CO_2_.

### 2.2. Plasmid Construction and Cell Transfection

The lentiviral plasmid encoding miR-29b and the negative control were designed and synthesized by Sheng Gong Bioengineering Co., Ltd. (Shanghai, China). A549 and NCI-H-1792 cells were grown to 20-30% confluence in a 6-well plate, and the medium was replaced with a 30- and 50-fold infection efficiency (MOI) lentivirus transfection enhancing solution. After 12 h, complete culture medium was used instead of culture for 72 h. Further, 1 *μ*g/ml puromycin was administered for 2 weeks to select the cells, and the cells were harvested for follow-up studies.

RETRACTED

### 2.3. Clonal Formation, Cell Proliferation, Invasion, and Scratching Experiments

In the invasion and wound healing test, transfected A549 cells or NCI-H-1792 cells were seeded on a 96-well plate, and the number of cells was measured by the cell counting CCK8 kit (Dojindo, Japan) at 1, 2, and 3 cell proliferation at 4 days according to the manufacturers' instructions. In the colony formation test, 300 transfected lung cancer cells were seeded on a 6-well plate and cultured for 14 days in DMEM with 10% FBS. The colonies were fixed with 95% ethanol and stained with 4 g/l crystal violet solution. The colonies containing more than 50 cells were counted. Cell invasion was detected in a Transwell chamber (BD Biosciences, San Jose, California, USA). Further, 600 *μ*l of complete medium was added to the lower chamber, the transfected cells were suspended in serum-free medium, and 200 *μ*l of cell suspension with 4∗104 cells was placed in the upper chamber. After 24 hours, the cells on the upper surface of the membrane were removed with cotton wool, and the cells were fixed in 95% ethanol and stained with 4 g/l crystal violet solution. The cells adhering to the bottom surface of the membrane were counted in five randomly selected areas. For the cell migration test, the cells were seeded on a six-well plate at 90% confluence and cultured overnight to allow the cells to adhere. Then, a 200 *μ*l pipette tip was used to scratch the cell layer, forming a wound along the center of each hole. Next, the wells were rinsed twice with phosphate buffered saline (PBS) to remove any loose cells, and fresh medium was added. Photographs were taken at 0 and 24 hours to assess the migration of cells to the wound. Each experiment was repeated three times.

### 2.4. Quantitative RT-PCR

TRIzol (Invitrogen; 15596018) reagent was used to extract total RNA from cells. Reverse transcription of miRNA or mRNA into cDNA with the reverse transcription kit (Thermo Scientific; K1691 or Promega A2800) was performed according to the manufacturer's instructions. RT-PCR (Invitrogen12594100 or Promega A6001) kit was used to detect the relative expression level of miR-29b. The RT-PCR reaction was performed with AB7500, and the reaction system and conditions were operated in accordance with the instructions. U6 was used as the internal reference control for miRNA detection, and GAPDH was used as the internal reference control for mRNA detection. The relative expression level of miRNA or mRNA was calculated using 2-△△ct.

RETRACTED

### 2.5. Luciferase Reporter Analysis

Briefly, 293T cells were seeded on a 24-well plate, and Lipofectamine 2000 (Invitrogen; 11668019) was used with FEM1B wild-type 3′-UTR (WT-3′-UTR) or mutant 3′-UTR (FEM1B MUT-3′-UTR) cotransfected with the luciferase reporter construct of miR-29b or miR-29b-NC. After the cells were incubated for 48 hours, they were washed with PBS and lysed with lysis buffer (Thermo Scientific; 87788). The dual luciferase detection was performed according to the instructions of the dual luciferase reporter kit (Thermo Scientific; 16186).

### 2.6. Apoptosis and Cell Cycle Detection

For trypsin digestion, the cells were resuspended to make a l × l06/ml cell suspension. An appropriate volume was taken, processed, and stained according to the apoptosis kit (Abcam; ab14085) and cycle detection kit (Invitrogen; A10798); then, a flow cytometer was used to measure the apoptosis or cycle of the sample.

### 2.7. Western Blot

The total protein was extracted from cells and tumor tissues, and the concentration of the extracted protein was determined by the BCA method. Further, 20 *μ*g/well was loaded and the protein was separated by SDS-PAGE. The separated protein was transferred to PVDF membrane, blocked with 5% BSA (Sangon), and the primary antibody was incubated overnight at 4°C. After incubating the secondary antibody, the ECL kit (Pierce) was used for color development and imaging. Western blot experiments were performed using the following antibodies: FOX01 (Abcam; ab55178), Sirt3 (Abcam; ab217319), AKT (Abcam; ab38449), p-AKT (Abcam; ab81283)), AKT (Abcam; ab8805), VEGF (Abcam; ab32152), GAPDH (Abcam; ab8245), and secondary antibody (Abcam; ab228530).

### 2.8. Prediction of the miRNA Target Interaction

At least two prediction databases, such as miRTarBase (version 6.0), DIANA, and TargetScan, were chosen to predict miRNA target genes.

### 2.9. Kaplan-Meier Survival Analysis

The data downloaded from TCGA database was used to analyze the survival rate of NSCLC patients. For miR-29b analysis, NSCLC patients were divided into two groups based on the miR-29b expression level: the miR-29b low expression group and miR-29b high expression group. Similarly, for the FEM1B analysis of NSCLC patients, according to their FEM1B expression levels, they were divided into two groups: FEM1B low and FEM1B high. The Limma software package was used to detect the miRNA and gene expression levels on the R platform. The purpose of setting the cut-off value was to separate the top 10% of patients with “miR-29b low” from 90% of patients with “miR-29b high” or to separate 10% of patients with “FEM1B high” from 90% of patients with “FEM1B low.” The patients were thus separated. The survival curve was estimated by the Kaplan-Meier method and compared with the log-rank test.

RETRACTED

### 2.10. Establishment of a Nude Mouse Xenotransplantation Model

Animal research was conducted in accordance with the guidelines of the animal care and the guidance of Committee of Meizhou People's hospital. In brief, 6-week-old BALB/c nude mice were subcutaneously injected with 6 × 106 cells stably expressing miR-29b or normal A549 cells. Mice were also injected with an empty vector on the right side. After 28 days, mice were sacrificed according to the standard procedures, and the tumors were taken and weighed. The volume of each tumor was calculated *b* × (*a* + *b*)/2 according to the formula *V* = *a*, where *a* and *b* are the length and width of the tumor measured by a vernier caliper, respectively.

### 2.11. Statistical Analysis

SPSS 19.0 (IBM, NY, USA) software was used for statistical analysis. All experiments were performed in triplicate; and the Kaplan-Meier method was used to analyze the overall survival rate, and the log-rank test was used to compare the differences in survival curves. *P* < 0.05 was considered statistically significant.

## 3. Results

### 3.1. The Expression of miR-29b Is Downregulated in Lung Cancer Cells

Through bioinformatics analysis, the expression of miR-29b in the tumor tissues and adjacent tissues of lung cancer patients was analyzed by the GEO data set, and results showed that miR-29b was downregulated in lung cancer tissues (Figure 1(a)). The reverse transcription-polymerase chain reaction (RT-PCR) was used to detect the expression of miR-29b in five NSCLC cell lines (A549, Calu-1, Calu-6, HCC827, and NCI-H-1792) and normal lung cell lines (Beas-2B). The results are shown in Figure 1(b). The expression level of miR-29b in NSCLC cells was lower than that in the normal lung cell line Beas-2B. Among the cell lines, A549 and NCI-H1792 had lowest expression levels of miR-29b. A549 and NCI-H-1792 cells were selected for follow-up tests. Survival analysis showed that lung cancer patients with high miR-29b expression had a higher long-term survival rate (Figure 1(c)) (http://www.oncomir.org/cgibin/cu-Stom SurvivalCurve.cgi).

### 3.2. Overexpression of miR-29b Inhibits the Growth of NSCLC Cells

The miR-29b overexpressing lentivirus was used to infect A549 and NCI-H-1792 cells, and the overexpression was verified by qPCR. Compared with the nontransfected group (NC group), the expression of miR-29b in the miR-29b overexpression group was significantly increased (*P* < 0.05). In order to further examine the effect of miR-29b on the proliferation of NSCLC cells, CCK8 and colony formation tests were used to verify this. Upregulation of miR-29b can significantly inhibit cell proliferation (*P* < 0.05) (Figure 2(b)). The results of the colony formation test showed that compared with the NC group, the number of colonies formed in the miR-29b group was significantly reduced (Figure 2(c)) (*P* < 0.05). The migration and scratch recovery ability of miR-29b group was significantly reduced (*P* < 0.05) compared with the control NC group (*P* < 0.05) (Figures 2(d) and 2(e)). Flow cytometry detection of cell apoptosis revealed that the apoptotic rates of miR-29b-A549 and miR-29b-NCI-H-1792 were 8.23 ± 1.02% and 8.22 ± 0.66%, respectively, which were significantly higher than those in the NC-A549 group (2.93 ± 0.22%) (*P* < 0.05) and NC-NCI-H-1792 group (5.23 ± 1.38%). The results of the cell cycle test showed that miR-29b could block cells in the G1-G2 phase and delay cell growth and proliferation (Figure 2(f)). These data confirmed that overexpression of miR-29b could significantly inhibit the proliferation, invasion, and metastasis of NSCLC cells in vitro.

RETRACTED

### 3.3. FEM1B Is a miR-29b Regulatory Target Gene

Bioinformatics prediction software TargetScan, miRTarBase, and DIANA were used to predict the possible target genes of miR-29b. All prediction results showed that FEM1B was the target gene of miR-29b. As shown in Figure 3(a), FEM1B 3+UTR contained a binding site for miR-29b.

In order to verify that FEM1B was the direct target gene of miR-29b, wild-type FEM1B WT-3′-UTR and mutant FEM1B MUT-3′-UTR luciferase reporter gene vectors were constructed. By cotransfecting miR-29b mimics with FEM1B WT-3′-UTR and FEM1B MUT-3′-UTR into 293T cells, as shown in Figure 3(b), FEM1B WT-3′-UTR reporter gene and miR-29b mimics. After 48 h of cotransfection, the luciferase activity was significantly reduced (*P* < 0.05), but there was no significant change in the luciferase activity when FEM1B MUT-3′-UTR and miR-29b mimics were cotransfected. The results indicate that miR-29b binds to FEM1B WT-3′-UTR, and FEM1B may be a direct target gene of miR-29b. In order to further verify that FEM1B is the direct target gene of miR-29b, RT-PCR and western blot (WB) were used to detect the expression of FEM1B in cells overexpressing miR-29b. Overexpression of miR-29b significantly reduced the expression level of FEM1B mRNA (*P* < 0.05) (Figure 3(c)) and downregulated the protein expression level of FEM1B (Figure 3(d)). This shows that miR-29b negatively regulates FEM1B, and FEM1B is the direct target gene of miR-29b.

### 3.4. miR-29b Inhibits the Proliferation, Invasion, and Metastasis of NSCLC Cells by Downregulating FEM1B

In order to further confirm that miR-29b can inhibit the proliferation, invasion, and metastasis of NSCLC cells, FEM1B, miR-29b, si-FEM1B, FEM1B, and FEM1B+miR-29b were transfected into A549 and NCI-H-1792 cells. Through RT-PCR detection, it was found that the downregulation of FEM1B gene expression and overexpression of miR-29b had similar functions, and both genes could inhibit the expression of FEM1B mRNA and protein (Figure 4(a)). CCK8, cell scratch, and invasion test results found that miR-29b and si-FEM1B could inhibit the proliferation, migration, and invasion of NSCLC cells (Figures 4(b)–4(e)). When FEM1B expression was restored in miR-A549 and miR-NCI-H-1792 cells, cell invasion and migration were increased, and the inhibitory effect of miR-29b on cells could be partially reversed. The experimental results show that FEM1B is the target gene of miR-29b, and miR-29b inhibits the growth and proliferation of lung cancer cells by downregulating FEM1B.

RETRACTED

### 3.5. miR-29b Inhibits the Growth of Mouse NSCLC Tissue

In order to further confirm the effect of miR-29b on tumor formation of NSCLC cells in vivo, miR-29b-A549 and miR-NC-A549 were subcutaneously inoculated into nude mice. The tumor volume and weight of mice in the miR-29b-A549 group were significantly smaller than those in the miR-NC-A549 group (*P* < 0.05) (Figure 5(a)), and tumor growth was inhibited.

In order to verify that miR-29b can also directly regulate FEM1B in vivo, RT-PCR and WB were used to detect the expression level of FEM1B in mouse tumor tissues and normal lung tissues. The expression of FEM1B mRNA in the miR-NC-A549 group was significantly higher than that in the miR-29b-A549 group (*P* < 0.05) (Figure 5(b)). The results showed that the expression of miR-29b in NSCLC tissue was negatively correlated with FEM1B. Detection of tumor necrosis factor-alpha (TNF-*α*), interleukin- (IL-) 10, and VEGF in tumor of mice by ELISA showed that the expressions of TNF-*α* (*P* < 0.05) and VEGF in the miR-29b group were lower than those in the NC-A549 group, and the expression of IL-10 was higher than that in the NC-A549 group. During the experiment, the mice were weighed once a week, and the results showed that with the growth of the tumor, the weight of mice in the NC-A549 group showed a downward trend, and the weight of mice in the miR-29 group showed a fluctuating change. The weight of mice in the group was greater than that of mice in the NC-A549 group. The results of this part of the experiment show that miR-29b can effectively inhibit the growth of NSCLC tumors and reduce the expression of inflammatory factors in peripheral blood.

### 3.6. Expression of miR-29b and Its Influence on Downstream Molecular Pathways

miRNA usually produces specific binding reactions with target genes, and it further regulates downstream molecules. In order to further verify the regulatory mechanism of miR-29b in the occurrence and development of lung cancer, we tested the expression levels of genes related to the FOX01/AKT signaling pathway downstream of miR-29b. As shown in Figure 6, when miR-29b was overexpressed in A549 and NCI-H-1792 cells, FEM1B and HIF-1*α*, Sirt1, and AKT gene expression levels were significantly reduced (*P* < 0.05), and FOXO1 and TNF-*α* levels were significantly increased (*P* < 0.05). The results of ELISA tested showed that TGF-*β* was significantly increased in the miR-29b group (*P* < 0.05), while the expressions of IL-6 and IL-10 were significantly lower than those in the miR-NC group (*P* < 0.05). When FEM1B was overexpressed, the expression levels of HIF-1*α*, Sirt1, and AKT genes were upregulated. The results of WB showed that when miR-29b was overexpressed, the FOXO1 levels were reduced in NSCLC cells, thereby the FOXO1 transcriptional activity was increasing and VEGF protein expression was decreasing. Besides, the expression levels of Sirt3 and Smad3 were also downregulated. These results indicate that when miR-29b is overexpressed, it can inhibit the phosphorylation of FOXO1 and increase the activity of FOXO1, thereby inhibiting activation of the FOXO1/AKT signaling pathway. When FEM1B was overexpressed, part of the inhibitory effect of miR-29b on the FOXO1/AKT pathway could be reversed. miR-29b can inhibit activation of the FOXO1/AKT signaling pathway by targeting FEM1B to inhibit the proliferation and invasion of NSCLC cells.

RETRACTED

## 4. Discussion

Literature studies have pointed out that miR-29b is closely related to tumor size, moisturization, grade, and degree of lymphatic metastasis. In this study, we explored the relationship between miR-29b and lung cancer and found that the expression level of miR-29b was significantly lower than that in adjacent tissues in NSCLC tissues. Bioinformatics analysis and fluorescein reporter gene experiment proved that FEM1B is the target gene of miR-29b, and the expression of FEM1B is negatively correlated with the expression of miR-29b in NSCLC cells. Similar to the effect of overexpression of miR-29b, silencing FEM1B can inhibit the growth and invasion of lung cancer cells. miR-29b may be used as a prognostic marker or a new target for lung cancer treatment.

A large number of studies have shown that miRNAs are closely related to the development of tumors, and a variety of miRNAs are involved in the occurrence and development of tumors. The mRNA expression of miR-29b is significantly decreased in breast cancer [20], muscle atrophy [21], colorectal cancer [22, 23], cardiac fibrosis [24], and diabetes [25–27]. In order to determine the clinical significance of miR-29b in tumors, Zhu et al. [28] identified the expression of miR-29b in cancerous tissues and adjacent tissues of 187 prostate cancer patients. They found that the miR-29b gene in adjacent tissues was higher than that in tumor tissues, and miR-29b is related to lymphatic metastasis, bone metastasis, and Gleason score. In order to explore the role of miR-29b in lung cancer cells, Xie et al. [29] inhibited its target gene strn4 and acted on NSCLC cells, and they found that it can inhibit the growth of NSCLC cells and promote lung cancer cell apoptosis. In order to further determine the role of miR-29b in lung cancer, bioinformatics methods were used to analyze the correlation between the expression of miR-29b and long-term survival in 427 lung cancer patients. The results showed that the expression level of miR-29b was low and long-term survival rate was also low. Thus, miR-29b may be involved in the occurrence and development of lung cancer, and it may become a potential target and treatment site for lung cancer diagnosis and prognosis evaluation.

RETRACTED

Studies have shown that miRNA may have two sidedness, and the expression level of miRNA in different diseases is not the same. The same miRNA can not only promote the occurrence of the disease but can also inhibit further progression of the disease. Upregulation of the miR-183 [30] expression level can effectively inhibit the metastasis and development of lung cancer. In lung cancer cells, miR-126 [31] can effectively inhibit cell proliferation, adhesion, and invasion, and it can reduce the expression of Crk protein. These two miRNAs inhibit the occurrence and development of lung cancer. In lung cancer, the expression levels of miR-34 [32, 33], miR-20b, and [34] miR-17 [35] are upregulated, which can promote the development of lung cancer and accelerate metastasis and invasion [36]. miR-29b has been confirmed to be significantly downregulated in breast cancer and prostate cancer, and overexpression of miR-29b can inhibit tumor cell proliferation, invasion, and metastasis, block tumor cells in the G1 phase, and accelerate their apoptosis. This result was verified in NSCLC cells. We constructed an overexpressing vector of miR-29b and transfected it into NSCLC cells and used flow cytometry to verify the apoptosis of NSCLC cells after overexpression. The results showed that it can effectively accelerate the apoptosis of NSCLC cells and can block the cell cycle in the G1-G2 phase. The results of Transwell assay revealed that overexpression of miR-29b can effectively inhibit the invasion and metastasis of NSCLC cells.

RETRACTED

The FEM1B gene is a homolog of FEM-1, which is involved in cell regulation, apoptosis, and glucose homeostasis in the body. Research by Subauste et al. [37] found that FEM1B gene expression is upregulated in mouse colon cancer models. Because of the difference in the microenvironment within the tumor, the expression of FEM1B is also different. In breast cancer, the expression of FEM1B is significantly downregulated, and FEM1B can promote the apoptosis of breast cancer cells. In this study, through bioinformatics prediction and in vitro verification of miR-29b target genes, the results showed that FEM1B and miR-29b have binding sites; hence, FEM1B is the target gene of miR-29b. When miR-29b was overexpressed, the gene expression and protein expression of FEM1B showed a downward trend, indicating that FEM1B is the direct target gene of miR-29b, and FEM1B can inhibit the expression of miR-29b.

## 5. Conclusion

In summary, the results of this experiment show that miR-29b is a tumor suppressor gene. Overexpression of miR-29b can target to inhibit the expression of FEM1B, further inhibit the activation of the FOXO1/AKT signaling pathway, inhibit the expression of VEGF, and promote the apoptosis of NSCLC cells.

## Figures and Tables

**Figure 1:** The expression of miR-29b is significantly reduced in non-small-cell lung cancer (NSCLC) cell proliferation, invasion, and metastasis of NSCLC cells in vitro. (a) GDS4794 from the GEO data set was collected, and paracancerous and lung cancer tumor samples were analyzed. (b) miR-29b expression was decreased in NSCLC cells. (c) The survival rate of lung cancer patients was analyzed using the data downloaded from The Cancer Genome Atlas (TCGA) database.

**Figure 2:** Overexpression of miR-29b inhibits the growth of NSCLC cells. (a) miR-29b expression was increased significantly after overexpression of miR-29b. (b) miR-29b inhibited the proliferation of A549 and NCI-H1792 cells. (c) miR-29b inhibited the formation of A549 and NCI-H-1792 cell clones. (d) miR-29b inhibited A549 and NCI-H-1792 cell invasion. (e) miR-29b inhibited A549 and NCI-H-1792 cell migration. (f) miR-29b promoted the apoptosis of A549 and NCI-H1792 cells. (g) miR-29b promotes apoptosis of A549 and nci-h1792 cells in G0-G1 phase. ^∗^*P* ≤ 0.05, comparison between the miR-29b group and miR-NC group.

**Figure 3:** FEM1B is a miR-29b regulatory target gene. (a) The predicted miR-29b binding site in the 3′-UTR of FEM1B and the mutated 3′-UTR of FEM1B, which were generated using the complementary sequence in the seed region of miR-29b. (b) miR-29b or NC and a luciferase vector encoding the WT or MUT FEM1B 3′-UTR were transfected into 293T cells, and the relative luciferase activity was measured. (c) Overexpression of miR-29b inhibited the expression of FEM1B mRNA in NSCLC cells. (d) Overexpression of miR-29b inhibited the expression of FEM1B protein in NSCLC cells; ^∗^*P* ≤ 0.05 compared with the NC-A549 group; ^#^*P* ≤ 0.05 compared with the NC-NCI-H-1792 group.

RETRACTED

**Figure 4:** Downregulation of FEM1B inhibits the proliferation, invasion, and metastasis of lung cancer cells. (a and b) FEM1B mRNA expression in NSCLC cells was significantly reduced after inhibiting FEM1B. (c) FEM1B was downregulated or miR-29b was overexpressed to inhibit the proliferation of A549 and NCI-H-1792 cells. (d and e) FEM1B was downregulated or miR-29b was overexpressed, and A549 cells inhibited the migration of NCI-H-1792 cells. (f) Downregulation of FEM1B or overexpression of miR-29b inhibited the invasion of A549 and NCI-H-1792 cells. ^∗^*P* ≤ 0.05, comparison between the miR-29b group and NC-group. ^#^*P* ≤ 0.05, comparison between the si-FEM1B group and NC group.

**Figure 5:** miR-29b inhibits the growth of NSCLC tissues in mice. (a) The change trend in mouse body weight. (b) miR-29b inhibited the growth of NSCLC tissue. (c) miR-29b inhibited the expression of FEM1B in mouse NSCLC tissue. (d) miR-29b inhibits TNF in tumor tissues of NSCLC mice and VEGF to promote the expression of IL-10. ^∗^*P* ≤ 0.05, comparison between the miR-29b group and NC-A549 group; ^#^*P* ≤ 0.05, comparison between the NC-A549 group and control group.

**Figure 6:** The effect of miR-29b expression on the downstream molecules in the signaling pathway. (a) RT-PCR showed that the expression level of HIF-1*α*, Sirt1, and AKT was decreased when miR-29b was overexpressed, while the level of TNF-*α* and FOX01 was increased when miR-29b was overexpressed. The siFEMB1 reversed this phenomenon. (b) The results of WB showed that when miR-29b was overexpressed, the expression levels of SMAD3 and Sirt3 were decreased and the TNF-*α*, VEGF, and FOX01 were increased. And the overexpression of FEM1B augments this phenomenon. (c) The expression ability of downstream molecular pathway factors in the supernatant of ELISA cells. ^∗^*P* ≤ 0.05, comparison between the miR-29b group and NC-A549 group; ^#^*P* ≤ 0.05, comparison between the si-FEM1B and NC-NCI-H1792 group.

## Data Availability

The data used to support this study is available from the corresponding author upon request.
